The article "Reduce Surface Electromyography Channels for Gesture Recognition by Multitask Sparse Representation and Minimum Redundancy Maximum Relevance" was published in 2021. Journal: J Healthc Eng.

# Reduce Surface Electromyography Channels for Gesture Recognition by Multitask Sparse Representation and Minimum Redundancy Maximum Relevance

**DOI:** 10.1155/2021/9929684

**Published:** 2021-05-27

**Authors:** Yali Qu, Haoyan Shang, Jing Li, Shenghua Teng

**Affiliations:** College of Electronic and Information Engineering, Shandong University of Science and Technology, Qingdao, China

## Abstract

Surface electromyography- (sEMG-) based gesture recognition is widely used in rehabilitation training, artificial prosthesis, and human-computer interaction. The purpose of this study is to simplify the sEMG devices by reducing channels while achieving comparably high gesture recognition accuracy. We propose a compound channel selection scheme by combining the variable selection algorithms based on multitask sparse representation (MTSR) and minimum Redundancy Maximum Relevance (mRMR). Specifically, channelwise features are first extracted to compose channel-feature paired variables, for which variable selection procedures by MTSR and mRMR are carried out, respectively. Then, we rank all the channels according to their occurrences in each variable selection procedure and figure out a certain number of informative channels by fusing these rankings of channels. Finally, the gesture classification performance using the selected channels is evaluated by the support vector machine (SVM) classifier. Experiment results validate the effectiveness of this proposed method.

## 1. Introduction

Surface electromyography (sEMG) is commonly used in clinical and engineering areas with the advantages of being noninvasive and convenient in signal acquisition. For example, sEMG reveals the information in diagnosing neuromuscular disorders [1, 2]. More generally, it may play important roles in the controlling of artificial assistance robots, arm prostheses, rehabilitation equipment, and some other instruments [3, 4].

Most of the related works have been carried out with sEMG of multiple channels to guarantee satisfactory recognition performance [5]. However, the increase of channels makes not only a high cost in engineering but also the great complexity of the sEMG devices and data processing burden. In addition, it could suffer from performance deterioration due to signal crosstalk [6, 7]. To overcome these problems due to multiple channels of sEMG, it is rewarding to select a reduced group of channels in a myoelectric control system. This is just the aim of our work which is to simplify the sEMG device by removing some redundant electrodes on the premise of desired classification performance.

## 2. Related Research and Motivation

Feature extraction is a routine procedure to describe the sEMG signals with a feature vector. Multitudinous features of time domain, frequency domain, and time-frequency domain have been widely applied in sEMG-based classification tasks. When multiple features are extracted for channels one by one, we could get a feature set with a quite large size (the number of features per channel times the number of channels). Hence, feature selection can be followed to reduce the feature redundancy and alleviate the curse of dimensionality, where metrics including scatter plot of features, statistical analysis, and recognition rate are applied to evaluate the effectiveness of features [8, 9], and feature search strategies including sequential forward selection (SFS), sequential backward selection (SBS), or bidirectional searching are adopted to find out the most informative features [10].

The article "Reduce Surface Electromyography Channels for Gesture Recognition by Multitask Sparse Representation and Minimum Redundancy Maximum Relevance" was published in 2021. Journal: J Healthc Eng.

Like feature selection in the point of lowering the feature size, channel selection will, in addition, remove those channels unnecessary or irrelevant to classify different gestures. In fact, channel selection is highly related to feature selection since features coming from all the channels are generally combined to create a set of channel-feature paired variables. Hence, channel selection can be the successor operation after feature selection, using the selected or fixed features.

To select useful channels from multielectrode, Nagata and his colleagues [11] used the recognition rate to evaluate each measurement channel and found out the best combination of channels by the Monte Carlo method. Huang et al. [12] applied SFS search strategy for expected channels where four kinds of time-domain features and an LDA classifier are used in the searching iteration. Khushaba and Al-Jumaily [13] also adopted a wrapper method, particle swarm optimization, in channel selection where the importance of subsets was measured using the error rates acquired from a multilayer perceptron trained with backpropagation neural network. Similar work by Oskoei et al. [14] employed a multiobjective genetic searching algorithm with the objective function of data separability index or classification rate. Besides, filter methods have also been applied to rank the channels, where the minimum Redundancy Maximum Relevance (mRMR) [15] was used by Liu et al. [16] and Gupta et al. [17], the Relief-F by Qu et al. [18], and the Markov random field (MRF) by Qu et al. [16] as well.

As shown in these aforementioned pieces of literature, channel selection could be conducted by fixing the feature subset. That means we cannot simultaneously select the best features and channels, which can be improved in the way as follows. Features and channels are combined to construct feature-channel pairs, leading to a hybrid feature-channel selection problem. By finding the least redundant and most informative group of feature-channel pairs among all the possible ones, the best channels should be the most repeated ones. In these aspects, some classic or modified ranking methods have been applied to select channel-feature variables, such as mRMR-FCO [19] and certain correlation-based or distance-based evaluation function in the work by Al-Angari et al. [20].

The article "Reduce Surface Electromyography Channels for Gesture Recognition by Multitask Sparse Representation and Minimum Redundancy Maximum Relevance" was published in 2021. Journal: J Healthc Eng.

Channel selection can follow a feature-channel filtering pipeline, but differing in specific ranking scores or search strategies. Our work is just under this kind of framework where we resort to the multitask sparse learning [21] together with mRMR filtering to pursue the discriminative sEMG channels across the classification for multiple gestures.

Since the classic least square regression model in sparse learning does not pursue the class-discriminative power of features, certain type of discriminative regularization terms is preferred to make up this limitation. Zhu et al. [22] put forward a group-sparsity-based least square regression framework integrating linear discriminant analysis and locality preserving projection. Similarly, to better capture the discriminative information among subjects, a multitask feature selection method was proposed to incorporate the intraclass and interclass Laplacian matrices [23]. But this kind of work will generally lead to a complicated optimization problem and most likely suffer from heavy computation cost.

Inspired by the works related to multitask sparse learning, for channel selection, we propose a channel selection method that combines the multitask sparse representation (MTSR) and mRMR algorithms. Instead of superimposing discriminative regularization terms in the MTSR framework, we evaluate the sEMG channels using the MTSR and mRMR, respectively, and then fuse their results to figure out the ideal channels in the end. The flowchart of this paper is shown in Figure 1.

## 3. Methods

### 3.1. Dataset and Evaluation Metrics

The sEMG dataset [24] contains thirty healthy normal-limbed subjects, who were kept relaxed and performed 7 distinct hand gestures including hand open, hand close, supination, pronation, wrist flexion, wrist extension, and rest. Eight surface electrodes were used for sEMG acquisition. In other words, we have signals with eight channels.

In this work, three classic measures, that is, precision, recall, and accuracy, are selected as indicators to evaluate the performance of gesture classification. These metrics are defined as follows:

(1) $$\begin{array}{c} \text{precision}=\frac{\text{TP}}{\text{TP}+\text{FP}}, \end{array}$$

(2) $$\begin{array}{c} \text{recall}=\frac{\text{TP}}{\text{TP}+\text{FN}}, \end{array}$$

(3) $$\begin{array}{c} \text{accuracy}=\frac{\text{TP}+\text{TN}}{\text{TP}+\text{FP}+\text{TN}+\text{FN}}, \end{array}$$

where TP, FP, TN, and FN are True Positive, False Positive, True Negative, and False Negative, respectively. An average of classification metrics in the experiments below will be obtained by 5-fold cross validation.

The article "Reduce Surface Electromyography Channels for Gesture Recognition by Multitask Sparse Representation and Minimum Redundancy Maximum Relevance" was published in 2021. Journal: J Healthc Eng.

### 3.2. Feature Extraction

To analyze the sEMG signal, a sliding window is adopted for the 8 channels. Totally 11 time-domain features, as listed in Table 1, are extracted which have been proved effective for myoelectric pattern recognition [16]. Thus, we have channel-feature paired variables with the size of 8 times 11.

*L* is the signal length, and *x*_*i*_ is the signal in an analysis window. SD is the standard deviation. *p* is the order of autoregressive model, *ε*_*i*_ is a white noise term, and the coefficients *a*_*p*_ are used as features.

### 3.3. Channel Selection Scheme

This study aims to reduce the sEMG channels by finding the least and best electrode locations to discriminate different hand motions. For channel-feature variables, we first perform a composite variable selection for the task of gesture motion recognition. Then, all channels will be ranked according to their occurrences in the selection of channel-feature variables, where MTSR and the mRMR variable ranking method are used, respectively. By fusing these two ranking results, we can finally get the ideal channels but with high recognition capability for hand gesture motions.

#### 3.3.1. MTSR-Based Variable Selection

Given a feature matrix *X* ∈ *R*^*d*×*n*^, where *d* and *n* are the numbers of features and samples, respectively, we also have a class indicator matrix *Y* ∈ *R*^*c*×*n*^ with the class number *c*. Since multiple response variables are included in the class indicator matrix *Y*, for each response variable, we can find a regression coefficient vector individually. By regularizing a least square regression model with an *ℓ*_2,1_-norm, the multiclass feature selection problem can be formulated as a sparse least square regression model as follows [21]:

(4) $$\begin{array}{c} \underset{W}{\min}\frac{1}{2}Y-W^{T}X_{F}^{2}+\lambda W_{2,1}, \end{array}$$

where  *W* ∈ *R*^*d*×*c*^ is a coefficient matrix for regression and the parameter *λ* is adopted to adjust the sparsity of *W*. By enforcing the group sparsity on the coefficient matrix with a *ℓ*_2,1_-norm, some rows in *W* will be zero. The first term in equation (4) controls the data fitting error, and the regularization parameter *λ* balances the relative importance of both terms. The larger *λ* results in more zero rows in the coefficient matrix. It can be assumed that the optimal solution would assign large weights to the important features and zero or small weights to the less important features.

The article "Reduce Surface Electromyography Channels for Gesture Recognition by Multitask Sparse Representation and Minimum Redundancy Maximum Relevance" was published in 2021. Journal: J Healthc Eng.

#### 3.3.2. mRMR Variable Ranking

The above MTSR method mainly focuses on the relationship between labels and features but ignores the relationship between features to some extent. Hence, we resort to mRMR algorithm to select features from a different perspective.

The mRMR criteria [15] aim to choose features that are mutually dissimilar to each other and marginally similar to the classification labels, ranking candidate component features based on compromise between relevance and redundancy. In this paper, we use mutual information to measure both redundancy and relevance.

Mutual information is defined as follows:

(5) $$\begin{array}{c} I\left(X;Y\right)=\iint^{}p\left(x,y\right)\log\frac{p\left(x,y\right)}{p\left(x\right)p\left(y\right)}\text{d}x\text{d}y, \end{array}$$

where *X* and Y denote two feature vectors and *p*(*x*, *y*) is the joint probabilistic density, while *p*(*x*) and *p*(*y*) are the marginal probabilistic densities. The goal is to find a subset *S* with *m* features, and the maximum relevance and the minimum redundancy are defined by equations (6) and (7):

(6) $$\begin{array}{c} \max\;D\left(S,c\right),\\ D=\frac{1}{\left|S\right|}\sum_{x_{i}\in S}I\left(x_{i};c\right), \end{array}$$

(7) $$\begin{array}{c} \min\;R\left(S\right),\\ R=\frac{1}{{\left|S\right|}^{2}}\sum_{x_{i},x_{j}\in S}I\left(x_{i};x_{j}\right)\;, \end{array}$$

where *x*_*i*_ is the *i*-th feature, *c* is the class variable, and *S* is the feature subset. The maximum relevance and the minimum redundancy are integrated by equation (8) or (9).

(8) $$\begin{array}{c} \max\Phi \left(D,R\right),\\ \Phi =D-R,\; \end{array}$$

(9) $$\begin{array}{c} \max\Phi \left(D,R\right),\\ \Phi =\frac{D}{R\;}. \end{array}$$

The incremental search method is used to find the approximate optimal feature. Supposing that we already have the feature set *S*_*m*−1_, the next step is to find the *m*-th feature from the feature set *X* − *S*_*m*−1_ maximizing Φ(*·*). The incremental algorithm optimizes the formula [15]

(10) $$\begin{array}{c} \max_{x_{j}\in X-S_{m-1}}\left[I\left(x_{j};c\right)-\frac{1}{m-1}\sum_{x_{i}\in S_{m-1}}I\left(x_{j};x_{i}\right)\right]. \end{array}$$

### 3.4. To Fuse the Channel Rankings

As stated above, we successively select the effective channel-feature pairs by MTSR and mRMR ranking method. Thus, we can get two groups of rankings for all channels according to their occurrences in the screened channel-feature variables. These two channel ranking methods work with different principles, but their corresponding results share common informative components even if they differ to a certain extent. We combine the two channel ranking results in the hope of avoiding decision faults to the utmost extent.

The article "Reduce Surface Electromyography Channels for Gesture Recognition by Multitask Sparse Representation and Minimum Redundancy Maximum Relevance" was published in 2021. Journal: J Healthc Eng.

## 4. Results

### 4.1. Channel Selection

Considering that 11 features are extracted for 8 channels each, we have 88 channel-feature paired variables in total for each analysis window. We apply the multiclass sparse representation model for the training data. According to equation (4), the parameter *λ* controls the sparsity of the coefficient matrix W, namely, the number of the screened channel-feature variables. The gesture recognition performance would be affected by features and classifiers we employed.

Let *λ* varies from 0.01 to 0.1, and channel-feature variables corresponding to nonzero rows of the coefficient matrix *W* are kept and fed to a support vector machine (SVM) classifier with radial basis function [25]. We hope to achieve a high recognition rate (accuracy is used in Section 4.1 and 4.3) while using only a few feature variables.

We make a comparison to show how to decide a proper value for *λ*. When *λ* varies from 0.01 to 0.1, the screened channel-feature number varies greatly but the recognition rate does not decrease too much. The changing of recognition rate and channel-feature number along with *λ* is shown in Figure 2. We can also see that a good balance between the recognition rate and channel-feature dimension can be achieved when *λ* equals 0.03. Accordingly, we will keep 36 channel-feature variables in the following channel selection procedure.

And for mRMR-based channel-feature selection, we also keep the top 36 variables which will be fused with the results of MTSR.

Table 2 lists the selected 36 channel-feature variables (features for each channel) by MTSR and mRMR, respectively. It is obvious that there is a certain difference between the screened results by these two methods. For instance, autoregressive features AR1 and AR2 play important roles in MTSR modal, being used by most channels. However, for mRMR, the two features only appear in channel ⑧. Therefore, we select channels based on channel utilization rather than analyzing the features. We count the number of times that any two channels occupy a common feature, namely, the number of features shared by a channel pair. The more frequently a channel is utilized, the more important the channel will be. The corresponding statistical results for MTSR and mRMR are shown in Tables 3 and 4 .

From Tables 3 and 4, we sort channels by the number of times which are used. For MTSR, the order is ②>③=⑧>⑤>⑦>①=④>⑥ and ①=⑤>⑧>③>⑦>②=⑥>④ for mRMR. By decision-making level fusion for channel selection, three channels ③, ⑤, and ⑧ are adopted for the subsequent gesture recognition.

The article "Reduce Surface Electromyography Channels for Gesture Recognition by Multitask Sparse Representation and Minimum Redundancy Maximum Relevance" was published in 2021. Journal: J Healthc Eng.

### 4.2. Feature Selection

Also based on the screened channel-feature variables by MTSR and mRMR, we list all the channels occupying a given feature (shown in Table 5). If a feature is shared by over half channels (>4), it will be selected for the gesture recognition task. Specifically, we have WL, AR1, and AR2 from MTSR-based results, and WL, IAV, SSI, and Kurtosis by mRMR. These six features, WL, IAV, SSI, Kurtosis, AR1, and AR2, will be fed into classifier in the following experiments.

### 4.3. Classification Performance Based on Channel and Feature Selection

According to Section 4.1, three channels (③, ⑤, and ⑧) are jointly selected by fusing MTSR and mRMR. We first compare the gesture classification performance using these three channels with those by MTSR or mRMR individually. For MTSR-based results, the top three channels are ②, ③, and ⑧, and the three channels ①, ⑤, and ⑧ are for mRMR. Their corresponding gesture recognition accuracies are shown in Figure 3. By combining MTSR and mRMR, channels ③, ⑤, and ⑧ are used and the average recognition rate is 98.68%, which is higher than that using channels ②, ③, and ⑧ or ①, ⑤, and ⑧ (the average classification accuracy is 95.59% for channels ②, ③, and ⑧ and 81.15% for channels ①, ⑤, and ⑧).

In addition, comparative experiments for gesture classification are carried out using two or four channels selected by different methods. When choosing two channels, we have channels ⑤ and ⑧ by fusing MTSR and mRMR. For MTSR-based method, the top two channels are ② and ③ or ② and ⑧; for mRMR, the selected two channels are ① and ⑤. The gesture classification accuracies are illustrated in Figure 4, where channels selected by jointly using MTSR and mRMR achieve the highest classification accuracy.

As for choosing four channels, channels ③, ⑤, ⑦, and ⑧ are selected by fusing MTSR and mRMR. For MTSR-based method, the top four channels are ②, ③, ⑤, and ⑧; for mRMR, the four channels are ①, ③, ⑤, and ⑧. Correspondingly, the gesture classification accuracies are drawn in Figure 5. It also verifies that channels selected by jointly using MTSR and mRMR achieve the highest classification accuracy.

### 4.4. Performance Evaluation and Comparison

To evaluate the performance of our method by fusing MTSR and mRMR for channel selection, comparative experiments are conducted in two aspects. Firstly, we further compare the proposed method with MTSR and mRMR in the task of channel selection. For the number of selected channels varying from 2 to 4, precision and recall for gesture classification corresponding to different method are listed in Table 6 where the selected channels are in square brackets.

The article "Reduce Surface Electromyography Channels for Gesture Recognition by Multitask Sparse Representation and Minimum Redundancy Maximum Relevance" was published in 2021. Journal: J Healthc Eng.

Compared with only 2 channels used, the recognition performance improves significantly when 3 channels are selected. It reveals that even 2 informative channels cannot capture enough information to distinguish different hand gestures in the experiment, where the best combination of 2 channels [5 8] is picked out by the proposed method. With more channels added in a certain range, the recognition performance will increase overall. In all cases, as shown in the table, our MTSR- and mRMR-fused methods outperform each of the two base methods alone.

Besides, a latest work proposed a mean Relief-F-based channel selection method (MRCS) [18]. Under the same experimental conditions including dataset and features, its classification performance is shown as the third row in Table 6. As for selecting four channels, the channel combination [1 3 5 7] is obtained by MRCS, and the corresponding classification rate is lower than our work here by selecting 3 channels or 4 channels. It should be noted that the classification performance can be further improved by using more informative features as demonstrated in the work [18], which will be our focus in the work later.

## 5. Conclusion

Recent developments in sEMG instrumentation have made it possible to record many channels from single or multiple muscles simultaneously. The current study combines MTSR and mRMR to process the channel-feature variables, aiming to reduce the channel number without degrading the gesture recognition performance.

For a gesture recognition task, sEMG dataset of 8 channels is recorded for 7 hand motions. Given the channel-features pairs obtained from time-domain features, the most informative channels are decided by the MTSR- and mRMR-combined variable selection method. The combination of MTSR and mRMR makes the selected variables not only reflect the relationship between labels and feature vectors but also try to meet the requirement of maximum relevance and minimum redundancy between vectors. Experimental results have verified the effectiveness of the proposed method.

It is worth noting that only time-domain features are extracted for sEMG signals in this paper. The channel selection operation is dependent on these features. More features generated in the frequency domain or time-frequency domain are to be used to test this feature/variable selection method in the coming work. In addition, this proposed method for feature selection can also be used in other pattern recognition and machine learning applications.

## Figures and Tables

**Figure 1:** Gesture recognition by reducing sEMG channels.

The article "Reduce Surface Electromyography Channels for Gesture Recognition by Multitask Sparse Representation and Minimum Redundancy Maximum Relevance" was published in 2021. Journal: J Healthc Eng.

**Figure 2:** Changes of recognition rate and channel-feature number when *λ* varies from 0.01 to 0.1.

**Figure 3:** The classification accuracies using three channels selected by different methods (channels ②, ③, and ⑧ are selected by MTSR, channels ①, ⑤, and ⑧ are selected by mRMR, and channels ③, ⑤, and ⑧ are jointly selected by the two methods).

**Figure 4:** The classification accuracies using three channels selected by different methods (channels ② and ③ and channels ② and ⑧ are selected by MTSR, channels ① and ⑤ are selected by mRMR, and channels ⑤ and ⑧ are jointly selected by the two methods).

**Figure 5:** The classification accuracies using three channels selected by different methods (channels ②, ③, ⑤, and ⑧ are selected by MTSR, channels ①, ③, ⑤, and ⑧ are selected by mRMR, and channels ③, ⑤, ⑦, and ⑧ are jointly selected by the two methods).

**Table 1:** Features extracted for each analysis window.

Acronym	Name	Number of features	Formula
WL	Waveform length	1	WL=∑_*i*=1_^*L*−1^|*x*_*i*+1_ − *x*_*i*_|
IAV	Integrated absolute value	1	IAV=∑_*i*=1_^*L*^|*x*_*i*_|
RMS	Root mean square	1	$\text{RMS}=\sqrt{\frac{1}{L}\sum_{i=1}^{L}x_{i}^{2}}$
SSI	Simple square integral	1	SSI=∑_*i*=1_^*L*^|*x*_*i*_|^2^
Kurtosis	Kurtosis	1	$\text{Kurtosis}=\frac{1}{L-1}\sum_{i=1}^{L}\left({\left(x_{i}-\bar{x}\right)}^{4}/{\text{SD}}^{4}\right)-3$
Skewness	Skewness	1	$\text{Skewness}=\frac{1}{L-1}\sum_{i=1}^{L}\left({\left(x_{i}-\bar{x}\right)}^{3}/{\text{SD}}^{3}\right)$
ZC	Zero crossing (threshold *T* = 10)	1	ZC=∑_*i*=1_^*L*−1^*φ*(*x*_*i*_, *x*_*i*+1_)
			$\varphi \left(x_{i},x_{i+1}\right)=\left\{\begin{array}{cc} 1, & x_{i}x_{i+1}<0,\left|x_{i}-x_{i+1}\right|>T,\\ 0, & \text{otherwise}, \end{array}\right.$
4AR	4th-order autoregressive model	4	*x*_*i*_=∑_*p*=1_^4^*a*_*p*_*x*_*i*−*p*_+*ε*_*i*_

**Table 2:** The selected 36 channel-feature variables by MTSR and mRMR. AR1∼AR4 are four coefficients in the fourth-order autoregressive model, respectively.

Channel	Features by MTSR	Features by mRMR
①	RMS, AR1, AR2, and AR4	WL, IAV, Kurtosis, SSI, and AR3
②	WL, Skewness, AR1, AR2, and AR3	WL, IAV, Kurtosis, and Skewness
③	WL, IAV, AR1, AR2, and AR3	WL, IAV, Kurtosis, and SSI
④	WL, IAV, AR1, and AR4	WL, IAV, and Kurtosis
⑤	RMS, Kurtosis, AR1, AR2, AR3, and AR4	WL, IAV, Kurtosis, SSI, and AR3
⑥	WL and Skewness	WL, IAV, SSI, and AR3
⑦	IAV, Skewness, AR1, and AR2	WL, IAV, Kurtosis, and AR3
⑧	WL, SSI, Kurtosis, Skewness, AR1, and AR2	WL, IAV, SSI, Kurtosis, Skewness, AR1, and AR2

**Table 3:** The number of times that two given channels occupy a common feature by MTSR (e.g., channel ① and channel ② share 2 features: AR1 and AR2). The best channels are in italics.

	Channel ①	Channel ②	Channel ③	Channel ④	Channel ⑤	Channel ⑥	Channel ⑦	Channel ⑧
Channel ①	—	2	2	2	4	0	2	2
Channel ②	2	—	4	2	3	2	3	4
Channel ③	2	4	—	3	3	1	3	3
Channel ④	2	2	3	—	2	1	2	2
Channel ⑤	4	3	3	2	—	0	2	3
Channel ⑥	0	2	1	1	0	—	1	2
Channel ⑦	2	3	3	2	2	1	—	3
Channel ⑧	2	4	3	2	3	2	3	—
Sum	14	*20*	*19*	14	*17*	7	16	*19*

The article "Reduce Surface Electromyography Channels for Gesture Recognition by Multitask Sparse Representation and Minimum Redundancy Maximum Relevance" was published in 2021. Journal: J Healthc Eng.

**Table 4:** The number of times that two given channels occupy a common feature by mRMR (e.g., channel ① and channel ② share 3 features: WL, IAV, and Kurtosis). The best channels are in italics.

	Channel ①	Channel ②	Channel ③	Channel ④	Channel ⑤	Channel ⑥	Channel ⑦	Channel ⑧
Channel ①	—	3	4	3	5	4	4	4
Channel ②	3	—	3	3	3	2	3	4
Channel ③	4	3	—	3	4	3	3	4
Channel ④	3	3	3	—	3	2	3	2
Channel ⑤	5	3	4	3	—	4	4	4
Channel ⑥	4	2	3	2	4	—	3	3
Channel ⑦	4	3	3	3	4	3	—	3
Channel ⑧	4	4	4	3	4	3	3	—
Sum	*27*	21	*24*	20	*27*	21	23	*25*

**Table 5:** Channels used by each feature.

Feature	Channels by MTSR	Selected	Channels by mRMR	Selected
WL	②③④⑥⑧	**√**	①②③④⑤⑥⑦⑧	**√**
IAV	③④⑦		①②③④⑤⑥⑦⑧	**√**
RMS	①⑤		–	
SSI	⑧		①③⑤⑥⑧	**√**
Kurtosis	⑤⑧		①②③④⑤⑦⑧	**√**
Skewness	②⑥⑦⑧		②⑧	
ZC	–		–	
AR1	①②③④⑤⑦⑧	**√**	⑧	
AR2	①②③⑤⑦⑧	**√**	⑧	
AR3	②③⑤		①⑤⑥⑦	
AR4	①④⑤		–	

**Table 6:** Comparison with different research methods.

Method	Channel	Recall	Precision	Channel	Recall	Precision	Channel	Recall	Precision
MTSR	[2 8]	83.69	84.59	[2 3 8]	95.30	95.60	[2 3 5 8]	96.82	97.18
mRMR	[1 5]	80.52	83.90	[1 5 8]	85.94	89.81	[1 3 5 8]	98.61	98.75
MRCS [18]	[1 5]	80.52	83.90	[1 5 7]	83.64	88.64	[1 3 5 7]	96.99	97.09
Our method	[5 8]	93.42	93.74	[3 5 8]	98.92	98.95	[3 5 7 8]	99.12	99.19

## Data Availability

The pattern recognition library is available at http://www.sce.carleton.ca/faculty/chan.
